# Application of Jianpi Xiaoai Recipe Combined with Cisplatin and Adriamycin in the Treatment of Endometrial Cancer and Its Effect on Disease Control Rate

**DOI:** 10.1155/2021/2258183

**Published:** 2021-09-28

**Authors:** Li Ding, Hongyu Li, Yuping Wang

**Affiliations:** ^1^Department of Gynaecology, People's Hospital of Rizhao, Rizhao 276826, Shandong, China; ^2^Department of Radiology, People's Hospital of Lixia District, Jinan 250013, Shandong, China; ^3^Department of Postpartum Rehabilitation, Zibo City Maternal and Child Health Care Hospital, Zibo 250031, Shandong, China

## Abstract

**Objective:**

To explore the application of Jianpi Xiaoai recipe combined with cisplatin and Adriamycin in the treatment of endometrial cancer (EC) and its effect on the disease control rate (DCR).

**Methods:**

The data of 120 EC patients treated in People's Hospital of Rizhao from February 2019 to February 2020 were retrospectively analyzed. They were equally split into experimental group and control group according to the order of admission. All patients were treated with neoadjuvant intra-arterial chemotherapy (continuous infusion of the uterine artery for 5 days before surgery, with 20 mg of cisplatin mixed with 2000 mg of normal saline and 10 mg of Adriamycin mixed with 500 ml of normal saline daily), while the experimental group was treated with Jianpi Xiaoai recipe at the same time to compare the short-term efficacy, immune function indexes, incidence of adverse reactions, and HEC-1-B (human endometrial adenocarcinoma cells) cell inhibition rates between the two groups.

**Results:**

The DCR and objective remission rate (ORR) in the experimental group were markedly higher compared with the control group (*P* < 0.05). The immune function indexes after treatment were remarkably better in the experimental group than in the control group (*P* < 0.05). Compared with the control group, the incidence of adverse reactions in the experimental group was notably lower (*P* < 0.05), while the HEC-1-B inhibition rates after treatment were obviously higher (*P* < 0.05).

**Conclusion:**

Jianpi Xiaoai recipe combined with cisplatin and Adriamycin can increase the HEC-1-B cell inhibition rate in EC patients, improve their immune function, reduce the possibility of adverse reactions, and enhance the therapeutic effect, which is worthy of clinical application and popularization.

## 1. Introduction

Endometrial cancer (EC) is an epithelial malignant tumor that occurs in the endometrium. According to the statistics from the American Cancer Society (ACS) in 2017, EC is the sixth most common female cancer, with the highest incidence in South America, Northern Europe, and Eastern Europe during 2006–2007. The risk of EC in Southeast Asia has surged in the past decade, with an increasing incidence in Japan, Singapore, and the Philippines year by year [1]. The EC incidence in China has also reached 10/100,000, becoming a female reproductive system malignant tumor only after cervical cancer [2]. Since the early symptoms of the disease are not obvious, and patients often suffer from symptoms such as vaginal bleeding, menstrual disorders, and lumbar-abdominal pain only after the disease progresses [3, 4], the diagnosis time of EC is often late and application of chemotherapy will cause serious adverse reactions due to gradually reduced immune function of patients [5, 6], affecting the overall therapeutic effect. Therefore, the selection of appropriate drugs to meet the maximum killing effect of cancer cells while minimizing its toxicity to normal cells has become the focus of the studies on chemotherapy.

Previous studies have shown that neoadjuvant intraarterial chemotherapy (cisplatin and Adriamycin) has a remarkable effect on cervical cancer [7], Nasioudis et al. applied it in the treatment of EC and found that this chemotherapy regimen can effectively reduce the mass volume and eliminate the possibility of subclinical metastasis [8]. A large number of international documents have confirmed that cisplatin and Adriamycin, like other antitumor drugs, kill cancer cells by inducing specific target molecule damage or dysfunction [9]. Although some studies have shown that they are safe and can reduce the incidence of complications in the subsequent surgery [10, 11], their effect on the incidence of adverse reactions in EC patients remains unclear. In recent years, Sugandha et al. found that based on the conventional chemotherapy regimens, dialectical application of Jianpi Xiaoai recipe can increase the disease control rate (DCR) of patients with advanced metastatic colorectal cancer and reduce the possibility of adverse reactions [11]. From the perspective of modern pharmacology, Jianpi Xiaoai recipe can also play a significant role in the treatment of EC because its components such as ginseng, *Astragalus*, poria, progesterone, and ginsenoside Rg3 can not only regulate the immune function of patients but also block the iron transport pathways of human endometrial adenocarcinoma cells (HEC-1-B), thus inducing apoptosis of cancer cells by inhibiting HEC-1-B and enhancing the therapeutic effect [12]. Therefore, this paper combined Jianpi Xiaoai recipe with cisplatin and Adriamycin to explore the application effect on EC patients, reported as follows.

## 2. Materials and Methods

### 2.1. Study Design

This retrospective study was conducted in People's Hospital of Rizhao from February 2019 to February 2020, aiming to explore the application of Jianpi Xiaoai recipe combined with cisplatin and Adriamycin in the treatment of endometrial cancer (EC) and its effect on the DCR.

### 2.2. Enrollment of Research Subjects

The data of 120 EC patients treated in People's Hospital of Rizhao from February 2019 to February 2020 were retrospectively analyzed. Patients were included according to the following criteria: (1) the patients were diagnosed with EC by preoperative fractional curettage pathology and postoperative pathological examination and met the diagnostic criteria in *Guidelines for the Diagnosis and Treatment of Endometrial Cancer (the 4*^*th*^*Edition)* [13]; (2) the patient had a good physical condition and could tolerate radiotherapy, chemotherapy, and surgical treatment; (3) the patients had no allergic reactions to the drugs involved in this study; and (4) the patients were expected to survive more than 3 months. Patients were excluded according to the following criteria: (1) the patients who were unable to communicate with others due to hearing impairment, language impairment, unclear consciousness, or mental illness; (2) the patients who quite the treatment halfway, died, changed the treatment regimens, and could not be followed up; (3) the patients complicated with serious heart, brain, liver, and kidney diseases or other malignant tumors; (4) the patients with incomplete clinical data; (5) the patients with low treatment compliance; (6) the patients in pregnancy and lactation; and (7) the patients who were treated in other medical institutions or participated in similar studies.

### 2.3. Steps

One hundred and twenty patients were enrolled in this study and were equally split into experimental group and control group according to the order of admission. On the day when the patients agreed to participate in the study, the research team collected their sociodemographic and clinical data and found no significant difference in the general data between the two groups after analysis (*P* > 0.05); see Table 1.

### 2.4. Moral Consideration

This study met the principles of the *Declaration of Helsinki* [14] and was approved by the hospital ethics committee. After enrollment, the research team explained the study purpose, significance, content, and confidentiality to the patients and asked them to sign the informed consent.

### 2.5. Exit Criteria

Judged by the research team, the patients with the following conditions were unsuitable to continuously participate in the experiment, and their medical records would be kept but not for data analysis: (1) the patients experienced adverse events or serious adverse events; (2) the patients had disease deterioration during the experiment; (3) the patients experienced severe comorbidities or complications; and (4) the patients who were unwilling to continue the clinical trial and requested for quitting the study during the experiment.

### 2.6. Methods

All patients were treated with neoadjuvant intraarterial chemotherapy, especially as follows: Seldinger technique was adopted to perform percutaneous puncture and intubation on one side of the femoral artery and insert a 5F catheter into the arteria iliaca communis. According to the tumor location and blood supply shown by the arterial angiography, the corresponding uterine artery was selected, and the catheter was retained to connect the infusion pump for continuous arterial infusion for 5 days. The patients daily received 20 mg of cisplatin (Qilu Pharmaceutical Co., Ltd.; National Medical Products Administration approval No. H20023460) mixed with 2000 mg of normal saline, and 10 mg of Adriamycin (Pfizer Wuxi Pharmaceutical Co., Ltd., National Medical Products Administration approval No. H20013334) mixed with 500 ml of normal saline, with an infusion rate of 110 ml/h. In addition, the patients were daily given 3000 ml of 5% glucose saline for hydration, making the patients' daily urine volume more than 2000 ml. The angiography was performed again after chemotherapy, and then extubation was performed. Surgery was performed at 3–4 weeks depending on the patients' condition.

At the same time, the experimental group was treated with Jianpi xiaoai recipe consisting of 15 g of ginseng, 15 g of radix curcumae, 15 g of poria, 20 g of astragalus, 20 g of oldenlandia, 20 g of sculellaria barbata, 6 g of fructus aurantii, 6 g of liquorice, 10 g of rhizoma pinellinae praeparata, and 5 g of epimedium. Radix ophiopogonis and dendrobium were added for patients with dry mouth; Fructus Amomi and bamboo shavings for patients with nausea and vomiting; fried *Evodia ruticarpa*, corydalis tuber, and Radix Paeoniae Alba for patients with gastrointestinal dysfunction; and angelica sinensis and spatholobus stem for those with blood deficiency. Jianpi Xiaoai recipe was decocted in warm water with one dose daily and was taken twice every day. Patients in the experimental group took the decoction for 2 months after the start of the neoadjuvant intraarterial chemotherapy.

### 2.7. Observation Criteria

1. General data: the general data extraction forms were established by the patients, including the in-patient number, name, age, pathological types, muscular infiltration, clinical staging, cytologic grades, menopause or not, marital status, and basic diseases.
2. Short-term efficacy: pelvic CT scan was performed in both groups at 1 month after treatment of the experimental group to evaluate the patient's short-term efficacy according to the response evaluation criteria in solid tumors (RECIST) [15] of the World Health Organization (WHO). The efficacy was classified as complete response (CR, complete endometrial withdrawal, stromal decidualization, and no endometrial hyperplasia or carcinoma), partial response (PR, reduced grades of endometrial lesions with residual cancer foci accompanied by gland degeneration and atrophy), stable disease (SD, no changes in endometrium with residual cancer foci and no endometrial degeneration and atrophy), and progression disease (PD, the presence of clear muscular infiltration or extrauterine lesions). Objective response rate (ORR) = CR + PR; DCR = CR + PR + SD.
3. Immune function indexes: 5 ml of fasting venous blood was extracted from patients in the morning before treatment (*T*_1_), 1 month after treatment (*T*_2_), and 2 months after treatment (*T*_3_). The level of immunoglobulin A (IgA) was detected by rate nephelometry (Shijiazhuang Hipro Biotechnology Corp., Hebei Medical Products Administration certificate no. 20162400132), and the NK, CD4^+^, and CD4^+^/CD8^+^ levels were detected by flow cytometry (ACEA BIO Hangzhou Co., Ltd.; Zhejiang Medical Products Administration certificate no. 20142400581).
4. Incidence of adverse reactions: adverse reactions after treatment were evaluated based on the manifestations and grading criteria of acute and subacute adverse reactions [14] of the WHO.
5. HUC-1-B cell inhibition rates: 5 ml of fasting venous blood was collected from the patients in the morning before treatment (*T*_1_), 1 month after treatment (*T*_2_), and 2 months after treatment (*T*_3_). Flow cytometry (ACEA BIO Hangzhou Co., Ltd.; Zhejiang Medical Products Administration certificate no. 20142400581) was adopted to detect the apoptosis of HUC-1-B cells.

### 2.8. Statistical Treatment

In this study, the data were processed by SPSS 20.0 software and graphed by GraphPad Prism 7 (GraphPad Software, San Diego, USA). This study included enumeration data and measurement data, tested by *X*^2^ and *t*-test. The differences were statistically significant at *P* < 0.05.

## 3. Results

### 3.1. Comparison of Patients' General Data

No remarkable differences in general data were observed between the two groups (*P* > 0.05); see Table 1.

### 3.2. Comparison of Patients' Short-Term Efficacy

The DCR and ORR in the experimental group were higher compared with the control group (*P* < 0.05); see Table 2.

### 3.3. Comparison of Patients' Immune Function Indexes

The immune function indexes after treatment were remarkably better in the experimental group than in the control group (*P* < 0.05); see Figure 1.

Note: in Figure 1, the abscissa from left to right represented before treatment (*T*_1_), 1 month after treatment (*T*_2_), and 2 months after treatment (*T*_3_). The lines with dots indicated the experimental group, and those with squares indicated the control group. # indicated *P* < 0.05.

Figure 1(a) shows IgA. No statistical difference in IgA at *T*_1_ was found between the two groups (2.64 ± 0.23 vs. 2.68 ± 0.24, *P* > 0.05). The IgA at *T*_2_ and *T*_3_ in the experimental group was markedly lower than that in the control group (1.68 ± 0.21 vs. 2.25 ± 0.25, 1.44 ± 0.18 vs. 2.04 ± 0.20, *P* < 0.001).

Figure 1(b) shows NK. No statistical difference in NK at *T*_1_ was found between the two groups (7.99 ± 0.45 vs. 8.10 ± 0.46, *P* > 0.05). The NK at *T*_2_ and *T*_3_ in the experimental group was markedly higher than that in the control group (11.13 ± 0.35 vs. 9.21 ± 0.12, 13.00 ± 0.48 vs. 11.10 ± 0.54, *P* < 0.001).

Figure 1(c) shows CD4^+^. No statistical difference in CD4^+^ at *T*_1_ was found between the two groups (34.58 ± 2.12 vs. 34.64 ± 2.13, *P* > 0.05). The CD4^+^ at *T*_2_ and *T*_3_ in the experimental group was remarkably higher than that in the control group (40.68 ± 3.10 vs. 36.57 ± 2.98, 44.68 ± 3.23 vs. 40.12 ± 3.24, *P* < 0.001).

Figure 1(d) shows CD4^+^/CD8^+^. No statistical difference in CD4^+^/CD8^+^ at *T*_1_ was found between the two groups (1.24 ± 0.12 vs. 1.23 ± 0.13, *P* > 0.05). The CD4^+^/CD8^+^ at *T*_2_ and *T*_3_ in the experimental group was remarkably higher than that in the control group (1.32 ± 0.24 vs. 1.20 ± 0.20, 1.35 ± 0.24 vs. 1.18 ± 0.21, *P* < 0.05).

### 3.4. Comparison of the Incidence of Adverse Reactions

Compared with the control group, the incidence of adverse reactions in the experimental group was notably lower (*P* < 0.05); see Table 3.

### 3.5. Comparison of HEC-1-B Cell Inhibition Rates

The HEC-1-B cell inhibition rates in the experimental group were remarkably higher compared with the control group (*P* < 0.05); see Figure 2.

Note: in Figure 2, the abscissa from left to right represented before treatment (*T*_1_), 1 month after treatment (*T*_2_), and 2 months after treatment (*T*_3_), and the ordinate represented the HEC-1-B cell inhibition rate (%). The black area was the experimental group and the gray area was the control group. # indicated *P* < 0.05.

No statistical difference in the HEC-1-B cell inhibition rates at *T*_1_ was observed between the two groups (6.98 vs. 6.96, *P* > 0.05).

The HEC-1-B cell inhibition rates at *T*_2_ and *T*_3_ in the experimental group were remarkably higher compared with the control group (60.24 vs. 40.47, 72.58 vs. 53.68, *P* < 0.001).

## 4. Discussion

EC is a female reproductive systemic malignant tumor with the incidence second only to cervical cancer [16], which is common in perimenopausal women. The early symptoms of EC are nonspecific, and patients may present with symptoms such as abnormal leukorrhea and lumbar-abdominal pain as the disease progresses, seriously threatening their life health. Although the EC incidence has remained high in the past decade, the academic community has not clarified its pathogenesis. Modern Western medicine believes that lifestyle changes, obesity, and hypertension are all high-risk factors for the EC occurrence [17], and the main clinical treatment methods are surgery and chemotherapy. However, surgical treatment alone cannot improve the 5-year survival rate of patients with infiltration of deep muscular layer and lymphatic space [18], so adjuvant chemotherapy is essential. Neoadjuvant intraarterial chemotherapy is often adopted in the treatment of gynecological malignancies such as cervical cancer, which has been proven to inhibit the proliferative activity of cancer cells and accelerate their apoptosis [19]. Although bilateral uterine arteries supply blood for the EC patients, the dominant lateral uterine artery was selected for continuous perfusion in some studies to prolong the contact time between drugs and cancer cells, thereby improving the killing ability of the drugs. To enhance the therapeutic effect, this study also chose unilateral perfusion. After treatment, the HEC-1- B cell inhibition rates of both groups were improved, indicating the efficacy of neoadjuvant chemotherapy in the EC treatment.

Some previous studies have shown that preoperative neoadjuvant intraarterial chemotherapy can reduce the incidence of postoperative complications [20], but the effect of this chemotherapy regimen on the adverse reactions of EC patients remains unclear. Therefore, reducing the incidence of adverse reactions of patients is the key to improve their quality of life. In recent years, the concept of holistic and dialectical treatment of traditional Chinese medicine (TCM) has achieved remarkable results in the treatment of malignant tumors. Many studies have confirmed that TCM can improve the immunity of patients with chemotherapy, reduce the destruction of chemotherapy to normal tissues, and curb the further spread of cancer cells [21]. The Jianpi Xiaoai recipe selected in this study is often used in the treatment of colorectal cancer and colon cancer, which can reduce the hematological and digestive tract adverse reactions of chemotherapy patients and improve the safety of chemotherapy [22]. Although the causes of EC and digestive system malignant tumors are different, TCM classifies them into categories of metrorrhagia and metrostaxis and accumulated diseases that are believed to be caused by dampness-heat and stasis, Qi-stagnation and blood stasis, and stagnation of liver Qi. The herbs in Jianpi Xiaoai recipe have significant effects on them because ginseng, as the principle drug in this recipe can replenish Qi to invigorate the spleen, percolate dampness and disinhibit water, and support the healthy energy; astragalus, the minister drug, can benefit Qi and supplement the deficiency; fructus aurantii and radix curcumae can promote Qi, oldenlandia can detoxify the body, rhizoma pinellinae praeparata can dispel dampness, and epimedium can strengthen spleen, in which the five drugs are the assistant drugs. The herbs in the recipe are properly mixed to play the role of removing stasis and eliminating stagnation.

From the perspective of modern pharmacology, ginseng is rich in ginsenoside Rg3 (CS-Rg3) that can effectively inhibit the main pathways for the survival of cancer cells, namely, the activity of PI3K and AKT, and then induce HEC-1-B apoptosis. Wang et al. have found that the combination of cisplatin and astragalus in human endometrial cancer cell line HEC-1-B can significantly improve the lethality of HEC-1-B in vitro, which is stronger than the sum of the two drugs alone, with the cell inhibition rate as 2.7 times that of cisplatin alone [23]. Therefore, the HEC-1-B cell inhibition rates in the experimental group after treatment were significantly higher compared with the control group (*P* < 0.05). In addition to HEC-1-B, the progesterone contained in *Astragalus* can also enhance the immune function of patients, so the experimental group had a lower incidence of adverse reactions and significantly better immune function indexes after treatment compared with the control group (*P* < 0.05). Moreover, poria can affect the expression of caspase-3 and Bcl-2, in which caspase-3 can lead to cell apoptosis while Bcl-2 can inhibit apoptosis. A study has shown that poria decoction for nude mice bearing EC can upregulate caspase-3 and downregulate Bcl-2 [24], indicating that poria have a positive effect on serum factor levels of EC patients. Therefore, in this study, the DCR and ORR in the experimental group were remarkably higher compared with the control group (*P* < 0.05). It is worth noting that the effect of the herbs in Jianpi Xiaoai recipe on the molecular level of EC patients needs to be further investigated.

In conclusion, Jianpi Xiaoai recipe combined with cisplatin and Adriamycin can increase the HEC-1-B cell inhibition rate in EC patients, improve their immune function, reduce the possibility of adverse reactions, and enhance the therapeutic effect, which is worthy of clinical application and popularization.

## Figures and Tables

**Figure 1:** Comparison of patients' immune function indexes ($\bar{x}\pm s$).

**Figure 2:** Comparison of HEC-1-B cell inhibition rates.

**Table 1:** Comparison of patient general data.

Items	Experimental group (*n* = 60)	Control group (*n* = 60)	*X*^2^/*t*	*P*
Age (years old)				
Range	28–70	27–68		
Average age	54.68 ± 5.21	54.56 ± 5.23	0.126	0.900

Pathological types				
Adenocarcinoma	52	50	0.261	0.609
Clear cell carcinoma	6	8	0.324	0.570
Adenoacanthoma	2	2	0.000	1.000
Muscular infiltration			0.135	0.714
Superficial muscular infiltration	26	28		
Deep myometrial invasion	34	32		

FIGO clinical stages				
I	12	14	0.196	0.658
II	32	30	0.134	0.715
II	16	16	0.000	1.000

Cytologic grades				
High differentiation	27	26	0.034	0.854
Middle differentiation	21	23	0.144	0.705
Poor differentiation	12	11	0.054	0.817

Menopause			0.035	0.853
Yes	35	36		
No	25	24		

Marital status			0.164	0.685
Married	42	44		
Unmarried/divorced/widowed	18	16		

Basic diseases				
Hypertension	20	18	0.154	0.695
Coronary heart disease (CHD)	12	11	0.054	0.817
Diabetes	12	12	0.000	1.000
Pulmonary diseases	13	10	0.484	0.487

**Table 2:** Comparison of patients' short-term efficacy [*n* (%)].

Group	CR	PR	SD	PD	ORR	DCR
Experimental group	24 (40.0)	24 (40.0)	10 (16.7)	2 (3.3)	48 (80.0)	58 (96.7)
Control group	16 (26.7)	20 (33.3)	14 (23.3)	10 (16.7)	36 (60.0)	50 (83.3)
*X* ^2^	2.400	0.574	0.833	5.926	5.714	5.926
*P*	0.121	0.449	0.361	0.015	0.017	0.015

**Table 3:** Comparison of the incidence of adverse reactions [*n* (%)].

Group	Experimental group (*n* = 60)	Control group (*n* = 60)	*X* ^2^	*P*
Leukopenia				
I-II	22 (36.7)	34 (56.7)	4.821	0.028
III-IV	10 (16.7)	22 (36.7)	6.136	0.013

Neutropenia				
I-II	18 (30.0)	30 (50.0)	5.000	0.025
III-IV	6 (10.0)	15 (25.0)	4.675	0.031

Thrombocytopenia				
I-II	5 (8.3)	20 (33.3)	11.368	0.001
III-IV	1 (1.7)	7 (11.7)	4.821	0.028

Decreased hemoglobin				
I-II	12 (20.0)	30 (50.0)	11.868	0.001
III-IV	2 (3.3)	8 (13.3)	3.927	0.048

Nausea and vomiting				
I-II	20 (33.3)	36 (60.0)	8.571	0.003
III-IV	10 (16.7)	22 (36.7)	6.136	0.013

Diarrhea				
I-II	12 (20.0)	24 (40.0)	5.714	0.017
III-IV	2 (3.3)	10 (16.7)	5.926	0.015

Anemia				
I-II	4 (6.7)	12 (20.0)	4.615	0.032
III-IV	0 (0.0)	6 (10.0)	6.316	0.012

Renal dysfunction				
I-II	0 (0.0)	4 (6.7)	4.138	0.042
III-IV	0 (0.0)	4 (6.7)	4.138	0.042

## Data Availability

Data to support the findings of this study are available on reasonable request from the corresponding author.
